RETRACTED

# The Relationship between VEGF-C, TAM, and Lymph Node Metastasis in Oral Cancer

**DOI:** 10.1155/2022/9910049

**Published:** 2022-06-28

**Authors:** Wei Yuan, Tao Tan, Ying Liu, Yingjie Du, Shengjuan Zhang, Junrong Wang

**Affiliations:** Oral and Maxillofacial Surgery, Hebei Eye Hospital, Xingtai, Hebei 054000, China

## Abstract

**Objective:**

To investigate the relationship between vascular endothelial growth factor-C (VEGF-C) and tumor-associated macrophages in oral cancer (TAMs) with lymph node metastasis.

**Method:**

From January 2018 to January 2022, 155 cases of oral cancer tissues and 165 cases of normal mucosal tissues were collected from oral surgical resection tissues or biopsy specimens in Hebei Eye Hospital. Oral cancer tissues were observed. The control group had normal mucosal tissues. The clinical and immune parameters were observed and the treatment of oral cancer is also briefly discussed.

**Results:**

The number of TAMs and the expression of VEGF-C in oral cancer tissues were significantly higher than those in normal tissues (*P* < 0.05). The lymphatic vessel density, the number of TAMs, and the expression of VEGF-C in the metastatic group were higher than in nonmetastatic group, and the lymphatic vessel density, the number of TAMs, and the expression of VEGF-C in the paracancerous tissues were higher than central tumor tissue in the metastatic group (*P* < 0.05). Univariate analysis showed that the number of TAMs was related to the histological stage and the pathological type of oral cancer (*P* > 0.05). The expression of VEGF-C was associated with the histological stage of oral cancer (*P* < 0.05). Compared with the immune function after different treatments, the contents of CD4+ in both groups was higher than before, and the combined treatment group was increased more than single treatment group (*P* < 0.05). The contents of CD3+ and CD8+ in the two groups were lower than before, and the combined treatment group was decreased higher than combined treatment group (*P* < 0.05).

**Conclusions:**

The number of TAMs and the expression of VEGF-C in oral cancer tissues are higher than normal tissues. The number of TAMs and the expression of VEGF-C are higher in patients with lymph node metastasis. TAMs and VEGF-C may play an important role in lymph node metastasis of oral cancer. Integrated traditional Chinese and Western medicine can improve the immune function of patients with oral cancer and may improve the therapeutic efficacy.

## 1. Introduction

Oral cancer, a malignant tumor of the head and neck region, is a malignant tumor that occurs in the patient's oral cavity and is one of the most common malignant tumors in clinical practice [1]. It can be divided into squamous cell carcinoma and adenocarcinoma according to pathological classification, and squamous epithelial cell carcinoma is the most common [2]. There are many causes of oral cancer, such as long-term alcohol consumption, smoking, lack of attention to oral hygiene, and long-term areca nut chewing that can lead to oral cancer [3, 4]. Gas, alcohol, and other components produced during smoking will stimulate the mucosa, leading to normal oral mucosal injury or even mutation. The destroyed mucosa or cells will be more sensitive to some carcinogens [5, 6]. Oral cancer is highly susceptible and its incidence ranks sixth among all cancers. There are 450,000 patients with oral cancer each year worldwide [7].

RETRACTED

Previous studies have shown that patients with oral cancer usually experience lymph node metastasis because there are many lymphoid tissues around the oral cavity, especially lymph nodes in the neck as well as lymph nodes in the face that are prone to metastasis [8, 9]. Studies have shown that there is a significant relationship between lymphatic vessel density in oral cancer and lymph node metastasis after operation. The measurement of lymphatic vessel density may have a certain value in predicting postoperative lymph node metastasis. The density of lymphatic vessels around nasopharyngeal carcinoma is closely related to lymph node metastasis. It is speculated that the density of lymphatic vessels around nasopharyngeal carcinoma is of great significance for cervical lymph node metastasis. Lymphatic vessel density is closely related to lymphangiogenesis in breast cancer and axillary lymph node metastasis in breast cancer. In recent years, with the continuous deepening study on cell growth factors, research has found that VEGF-C is one of the growth factors closely related to a variety of malignant tumors, and its expression level is closely related to the occurrence and metastasis of hundreds of tumors such as lung cancer and gastric cancer [10, 11]. The correlation between VEGF-C and lymph node metastasis of oral cancer can be an important direction to explore. Moreover, many studies have revealed that tumor-associated macrophages play a nonnegligible role in the occurrence, growth, and metastasis of tumors. It is speculated that macrophages may promote the expression of vascular endothelial growth factor, which makes tumors metastasize in patients.

At present, there are many treatments for oral cancer. Western medicine includes chemotherapy and surgery. But long-term chemotherapy will also cause toxic and side effects to patients and affect the immune function of patients [12]. Traditional Chinese medicine (TCM) believes that oral cancer is caused by the dysfunction of the three viscera of the heart, spleen, and stomach, which requires tonifying the patient's five viscera qi and blood. A variety of traditional Chinese medicines can play a role in enhancing the immune function of patients, tonifying qi and elevating yang, detoxifying, blocking cancer, and treating cancer [13].

RETRACTED

In summary, it is very important to explore the mechanism of lymph node metastasis and oral cancer treatment options. In this study, we conducted a retrospective study of patients with oral cancer. The relationship between VEGF-C, TAMs and lymph node metastasis was explored, compare the changes of immune function after treatment with integrated traditional Chinese and Western medicine and Western medicine. It may find an effective treatment plan to provide a reference for clinical practice.

## 2. Materials and Methods

### 2.1. Study Design

From January 2018 to January 2022, 155 cases of oral squamous cell carcinoma and 165 cases of normal mucosa were retrospectively analyzed. There was no difference in the baseline of patients (*P* > 0.05). Informed consent was obtained from all patients. The study was approved by the Ethics Committee of Hebei Eye Hospital (No. HBE201821). All participants underwent a complete medical history and clinical examination. The surgical sections or biopsy specimens collected from patients with oral diseases were confirmed to meet the experimental requirements by pathological examination.

### 2.2. Observation Indicators

1. Macrophages are counted by randomly observing 10 high-power fields, counting the number of macrophages in each field, and calculating their average value is the number of macrophages in this tissue. The expression of VEGF-C was calculated using HPIAS-2000 computer image analysis software.
2. Immunohistochemical staining was performed using D2–40 specific markers to detect the density of lymphatic vessels contained in the tissue and reflect the degree of lymph node metastasis in the tissue by the size of lymphatic vessel density.
3. Univariate logistic regression was used to analyze the relationship between relevant parameters and the number of TAMs and the expression of VEGF-C.
4. 156 patients with oral cancer were randomly divided into combination therapy group (75 cases) and single therapy group (80 cases), and the combination therapy group was treated with integrated traditional Chinese and Western medicine (surgery and continuous arterial infusion chemotherapy method binding Tongluo Jiedu Method of TCM). The single treatment group was treated with Western medicine (surgery and continuous arterial chemotherapy). Venous blood was collected from the two groups before and 2 weeks after treatment. The contents of CD3+, CD4+, and CD8+ T cells were measured by a cell instrument. The changes of related immune function were observed and compared between the two groups before and after treatment.

RETRACTED

#### 2.2.1. Notes

1. Tongluo Jiedu method drug ingredients: dandelion, diffusa, astragalus, nine fragrances, leonurus, *Salvia miltiorrhiza*, bean root, fried jujube kernel, curcuma, ophiopogon, paeony, and coix seed.
2. The normal reference values were 67.84 ± 075 for CD3+, 35.14 ± 3.69 for CD4+, and 27.49 ± 1.68 for CD8+.

### 2.3. Inclusion and Exclusion Criteria

Inclusion criteria were as follows: (1) patients who met the relevant diagnostic criteria of oral cancer in Oral Science, diagnosed as oral cancer; (2) patients with no other malignant tumors; (3) patients with normal liver and kidney function; (4) patients with normal immune function; exclusion criteria were as follows: (1) patients without informed consent; (2) patients who were allergic to the traditional Chinese medicine used in the experiment; (3) patients with distant metastasis; and (4) patients with abnormal physical condition who cannot receive continuous arterial infusion chemotherapy.

### 2.4. Statistical Analysis

SPSS 25.0 software was used to analyze the data. The clinical data (measurement data) were expressed as mean ± standard deviation (*x* ± *S*). One-way ANOVA was used for comparison between groups. The *t* test was used for intragroup comparison, and the analysis of variance was used for the comparison between groups. The enumeration data were expressed by the number of cases (percentage), and the *χ*2 test was used. <0.05 means the difference is statistically significant (*P* < 0.05).

## 3. Results

There were 155 patients in the observation group and 165 patients in the control group. There were 92 males and 63 females in the observation group, aged 18–76 years, with an average age of 58.7 ± 8.5 years and a BMI of 25.03 ± 2.11; there were 71 males and 94 females in the control group, aged 25–73 years, with an average age of 59.0 ± 7.8 years and a BMI of 24.93 ± 2.32. There was no difference in the condition and other general data of the selected patients (*P* > 0.05). See Table 1 for details.

### 3.1. The Number of TAMs and the Expression of VEGF-C

The number of TAMs and the expression of VEGF-C in the observation group were higher than in the control group (*P* < 0.05, Table 2).

### 3.2. The Relationship Lymphatic Vessel Density, TAMs, and VEGF-C between Lymph Node Metastasis

The lymphatic vessel density, the number of TAMs, and the expression of VEGF-C in patients in the lymph node metastasis group were higher than in patients in the lymph node metastasis group. In patients with lymph node metastasis, the lymphatic vessel density, the number of TAMs, and the expression of VEGF-C in paracancerous tissue were higher than in tumor tissue (*P* < 0.05), while the density of lymphatic vessels, the number of TAMs, and the expression of VEGF-C in tumor tissue were not significantly different from those in paracancerous tissue (*P* > 0.05; Table 3).

RETRACTED

### 3.3. The Relationship between Related Parameters and the Number of TAMs and VEGF-C Expression

The number of TAMs was related to the histological stage of oral cancer and the pathological type of oral cancer (*P* > 0.05), but not to the patient's gender, age, or duration of oral cancer (*P* < 0.05), and the expression of VEGF-C was related to the histological stage of oral cancer (*P* < 0.05), but not to the patient's gender, age, duration of oral cancer, or pathological type of oral cancer (*P* > 0.05, Table 4).

### 3.4. Comparison of Immune Function after Different Treatments

Before treatment, the contents of CD4+ were lower than the normal values, and the contents of CD3+ and CD8+ were higher than the normal values in both groups, but the difference was not statistically significant (*P* > 0.05). After treatment, the content of CD4+ in both groups was higher than before, and the combined treatment group had a higher increase than the single treatment group (*P* < 0.05). The contents of CD3+ and CD8+ in the two groups were lower than before, and the combined treatment group decreased higher than the single treatment group (*P* < 0.05, Table 5).

## 4. Discussion

Oral cancer, as a malignant tumor with a high incidence, accounts for 1% of systemic malignant tumors and has strong lymph node metastasis, which seriously threatens the health and life of patients [14]. Macrophages are inflammatory cells and derived from monocytes, which are also known as tumor-associated macrophages because of their important role in tumor development [5]. In the early stage of oral cancer, macrophages inhibit angiogenesis and arouse the body's immunity. With the further development of oral cancer, regulated by the body environment as well as cellular growth factors, the function of macrophages changes, promoting the proliferation of tumor cells and providing help for further invasion and metastasis of oral cancer cells [15, 16]. One of the cellular growth factors that affect macrophages to exert their normal function is VEGF-C in oral cancer tissues [5]. VEGF-C, the first cellular growth factor discovered to be able to promote lymphangiogenesis, is isolated and purified from human prostate cancer cells and plays a role in a number of physiological activities in the human body [17]. Previous studies have confirmed that VEGF-C is closely related to lymph node metastasis. On the one hand, VEGF-C is abundantly expressed in macrophages, which not only changes the physiological function of macrophages but also promotes the proliferation of macrophages and promotes the formation of blood vessels and lymph nodes through the cytokines produced by macrophages; on the other hand, the expression level of VEGF-C in the paracancerous tissues is higher than tumor tissues, accelerating the binding rate of VEGF-C to the specific receptors on the surrounding normal lymph node cells and inducing the proliferation and migration of lymph nodes, resulting in further deterioration of the patient's condition [18–21].

RETRACTED

This study showed that the number of TAMs and VEGF-C expression in oral cancer tissues were higher than in normal tissues. These results indicate that VEGF-C and TAMs are abundantly expressed in oral cancer tissues. The density of lymphatic vessels, the number of TAMs and the expression of VEGF-C in the lymph node metastasis group were higher than those in the nonmetastasis group, and the density of lymphatic vessels, the number of TAMs and the expression of VEGF-C in paracancerous tissues in the metastasis group were higher than tumor tissues. With the development of oral cancer, VEGF-C affects macrophages to play a normal function, promotes the proliferation of tumor cells, and helps oral cancer cells to further invade and metastasize [22, 23]. Higher TAMs numbers and higher expression levels of VEGF-C lead to more lymph node metastasis. The univariate analysis showed that the number of TAMs was related to the histological stage and pathological type of oral cancer, and the expression level of VEGF-C was related to the histological stage of oral cancer. CD3 +, CD4+, and CD8+ belong to T lymphocyte subsets, which can effectively participate in and regulate the body's immunity and effectively respond to the body's immune situation of patients. After treatment, the immune function of the two groups increased more than before, and the degree of increase in the combined treatment group was higher than in the single treatment group. The content of CD3+ and CD8+ in both groups were lower than before, and the decrease was more significant in the combined treatment group. It shows that integrated traditional Chinese and Western medicine treatment can improve the immune function of patients with oral cancer, which may improve the therapeutic efficacy. Previous studies have also shown that integrated traditional Chinese and Western medicine treatment improves the therapeutic efficacy of patients with oral cancer, improves the patient's immunity, and brings new hope for the treatment of patients with oral cancer [19, 24, 25]. Traditional Chinese medicine has a very good therapeutic position in the treatment of breast cancer, gastric cancer, and other diseases. The cooperation and complementarity of traditional Chinese and Western medicine can improve the curative effect.

RETRACTED

In summary, oral cancer is harmful to people. The number of TAMs and VEGF-C expression in oral cancer tissues is higher than normal tissues. The number of TAMs and VEGF-C expression in patients with lymph node metastasis is high. Macrophages and VEGF-C may play an important role in lymph node metastasis of oral cancer. Integrated traditional Chinese and Western medicine treatments can improve the immune function of patients with oral cancer and may improve the therapeutic efficacy.

## Figures and Tables

**Table 1:** Baseline characteristics.

	Observation group (*N* = 155)	Control group (*N* = 165)
Gender (male/female)	92/63	71/94
Age (*x* ± *S*, years)	58.7 ± 8.5	59.0 ± 7.8
Weight (kg)	64.24	26.58
BMI (*x* ± *S*, kg/m^2^)	25.03 ± 2.11	24.93 ± 2.32

**Table 2:** Number of TAMs and expression of VEGF-C in tissues.

Group	Number of TAMs	Expression rate of VEGF-C (%)
Observation group (*n* = 155)	90.53 ± 1.63	12.12 ± 2.16
Control group (*n* = 165)	88.47 ± 1.85	11.32 ± 2.44
*T*	10.542	3.098
*P*	<0.001	0.002

**Table 3:** Relationship between lymph node metastasis and lymphatic vessel density, number of TAMs, and VEGF-C expression.

Group	Lymphatic vessel density		TAMs number		VEGF-C expression (%)	
	Paracancerous tissue	Tumor tissue	Paracancerous tissue	Tumor tissue	Paracancerous tissue	Tumor tissue
Lymph node metastasis group (*n* = 52)	8.82 ± 1.93a	7.01 ± 1.72	88.46 ± 2.41a	86.63 ± 2.50	11.89 ± 2.25a	10.67 ± 2.62
Nonmetastatic group (*n* = 103)	7.51 ± 1.80	6.27 ± 1.84	86.25 ± 2.91	85.37 ± 2.18	10.97 ± 2.42	9.54 ± 2.05
*T*	4.175	2.415	4.718	3.232	2.287	2.944
*P*	<0.001	0.017	<0.001	0.002	0.024	0.005

Note: ^a^*P* < 0.05.

**Table 4:** Relationship between TAMs number, VEGF-C expression, and related parameters.

		TAMs number	*P* value	VEGF-C expression	*P* value
Sex					
Male	92	83.26 ± 1.39	0.822	7.54 ± 1.61	0.742
Female	63	83.31 ± 1.30		7.46 ± 1.27	
Age					
18–32 years	34	83.18 ± 2.05	0.799	8.38 ± 2.20	0.740
32–46 years	60	83.30 ± 1.97		8.13 ± 1.45	
46–60 years	61	83.75 ± 1.07		8.20 ± 1.71	
Disease course					
1–3 years	29	83.12 ± 1.93	0.825	9.01 ± 1.63	0.847
3–5 years	75	83.66 ± 2.02		8.64 ± 0.13	
5–7 years	89	83.86 ± 2.16		7.22 ± 1.25	
Histological staging					
Stage 1, 2	53	83.50 ± 1.88	0.004	10.25 ± 1.97	0.031
Stage 3	62	86.21 ± 2.35		11.36 ± 0.55	
Stage IV	40	89.67 ± 2.79		12.78 ± 1.04	
Type of oral cancer					
Tongue cancer	57	86.29 ± 1.87	0.025	7.98 ± 1.28	0.661
Carcinoma of floor of mouth	68	87.32 ± 1.50		7.61 ± 1.52	
Carcinoma of maxillary sinus	30	89.45 ± 2.07		8.42 ± 1.37	

RETRACTED

**Table 5:** The effect of Western medicine treatment and integrated traditional Chinese and Western medicine treatment on immune function.

Group	CD3+ (%)		CD4+ (%)		CD8 (%)	
	Before treatment	After treatment	Before treatment	After treatment	Before treatment	After treatment
Combined treatment group (*n* = 75)	69.47 ± 2.32	67.42 ± 2.70a	30.13 ± 7.32	33.27 ± 2.66a	32.64 ± 8.72	29.31 ± 1.62a
Single treatment group (*n* = 80)	70.01 ± 1.83	69.77 ± 1.60a	29.37 ± 6.94	31.93 ± 3.96a	33.28 ± 8.65	32.75 ± 1.74a
*T*	1.618	6.669	0.664	2.456	0.459	12.717
*P*	0.108	<0.001	0.508	0.015	0.647	<0.001

Note: ^a^*P* < 0.05.

## Data Availability

The data used to support the findings of this study are available from the corresponding author upon request.
